This article has been retracted.

# CYP1B1 Gene Polymorphism Based on Health Monitoring and Nursing Methods after Minimally Invasive Surgery for Lung Cancer

**DOI:** 10.1155/2022/7042014

**Published:** 2022-09-07

**Authors:** Chunyan Liu, Bo Liu, Xia Han, Yanfen Zhang

**Affiliations:** Xingtai People's Hospital, Xingtai 054001, Hebei, China

## Abstract

The rapid development of science and technology has become an indispensable part of human life. Minimally invasive lung cancer surgery, that is, thoracoscopic surgery and da Vinci robotic surgery, has many advantages over previous surgeries, there is no need to make a large incision in the chest, the patient after such surgery, and recovery is also better and can also reduce the incision of the operation. Therefore, with the rapid development of science and technology today, how to detect changes in patients' health and establish an intelligent health monitoring system has become a development trend. This paper proposes to apply health monitoring in CYP1B1 gene polymorphism and nursing after clinical treatment of minimally invasive lung cancer surgery, after analyzing the society's demand for real-time health monitoring in this paper. It also studies the health monitoring system based on the advantages of smart phones. The system is suitable for the Android operating system and can monitor the temperature, weight, and other data of the human body. The experimental results show that the data value of the information displayed by the android software has a high degree of matching with the measured value, which basically keeps floating around 80, and the data consistency is strong.

## 1. Introduction

At present, with the rapid development of science and technology, intelligent health monitoring is rapidly popularized in people's daily life. Using smart phones to view people's physiological parameters will greatly promote the development of home intelligent monitoring systems. It is very important to establish smart home health monitoring systems such as wearable monitoring systems and remote medical monitoring. Intelligent health medical monitoring is the trend of future health development. Colleagues and human intelligent health monitoring system can realize the real-time monitoring of the detected person's blood pressure, body temperature, heart rate, heart sound, pulse, etc.; the equipment flexibility is good; the scalability is strong, portable, and easy to use; and at the same time, a number of physiological parameters of the human body can be collected, so as to conduct comprehensive analysis and judgment of data, and obtain the health status of the detected person.

Intelligent health monitoring uses wearable sensors to collect the physiological parameters of the guardian in real time. It transmits the collected physiological information to guardians and medical staff for modern communication through computer network technology. The patient's physiological parameters are monitored through the wearable physiological monitoring part. After the treatment, it sends the monitoring results to the mobile phone software on the application side. It monitors the abnormal conditions of patients in real time and sends SMS reminders in time. The mobile app can also send web pages to a remote monitoring server. In order to realize the telemedicine service of medical staff to patients, it has important application value in the future human intelligent life.

The innovation of this paper is that (1) it applies intelligent monitoring to CYP1B1 gene polymorphism and nursing methods after minimally invasive surgery for lung cancer, which is innovative to a certain extent. (2) It provides follow-up testing for the care of patients with CYP1B1 gene polymorphism and lung cancer after minimally invasive surgery and clinical treatment to ensure full recovery. In summary, the findings illustrate that the CYP1B1 gene polymorphisms are of interest in the study of minimally invasive surgery for lung cancer.

## 2. Related Work

With the development of science and technology, health detection systems have penetrated into all aspects of people's lives. More and more scholars are studying it. Adam et al. presented a comprehensive overview of structural health monitoring (SHM) using wireless sensor networks [1]. Mizoue developed a semi-automatic image analysis system CROCO in order to evaluate canopy condition in forest health monitoring [2]. Gui et al. proposed three optimization algorithms for damage detection based on support vector machines. The two different characterization methods it uses have also demonstrated that proper characterization is critical for improving sensitivity in detecting damage and assessing structural health. However, a support vector machine is a binary classification model whose basic model is a linear classifier defined with the largest interval in the feature space [3]. Nia et al. quantified the energy and storage requirements of a continuous personal health monitoring system using eight biomedical sensors. His analysis shows that there is a large gap between the long-term continuous monitoring of energy and storage needs and the capabilities of current equipment [4]. To monitor local critical regions of structures, impedance-based methods utilize the high-frequency impedance responses sensed by piezoelectric sensors as local dynamic features. Huynh et al. presented the current status and future challenges of impedance-based structural health monitoring [5]. With the rapid development of sensing technologies such as radio frequency identification and sensors, as well as the integration of information technologies such as wireless communication and the Internet, the Internet of Things is becoming an important technology for monitoring systems. C reviews and introduces a structural health monitoring (SHM) framework utilizing IoT technology for intelligent and reliable monitoring. It specifically introduces the technologies involved in the implementation of IoT and SHM systems and data routing strategies in the IoT environment. SHM is a multidisciplinary interdisciplinary field that involves the use of a large number of sensors and instruments to automatically sense structural loads and responses, and then to make health diagnoses of structures based on the collected data [6]. The downside of these studies, however, is that the considerations are not comprehensive enough. It has great uncertainty, and its practicability needs further investigation.

## 3. Intelligent Health Monitoring and Related Methods

### 3.1. Related Technologies of Intelligent Health Monitoring System

The hardware controller of this article is the STM32F105RBT6 of the ARM9 series. It uses wireless WiFi module to realize the parameter transmission of physiological parameter information. The software is using Android to develop mobile monitoring terminal and PC-side Java EE server program [7, 8].

#### 3.1.1. Overall Design Scheme of the System

The system consists of four parts: wearable detection module for physiological parameters, processing of main controller and intelligent medicine box module for drug management, smart phone software monitoring module, and remote monitoring server module. Physiological parameters wearable detection module is a kind of wearable detection instrument designed according to physiological structure parameters, the main controller processing and drug management intelligent pill box module are suitable for controlling the module of the agent, the smart phone software monitoring module is the use of smart phone detection module, and remote monitoring server module refers to the use of smart phone software system, to achieve the purpose of remote monitoring. The overall structure of the system is shown in Figure 1.

#### 3.1.2. Smartphone Control Terminal Interface Architecture

The purpose of this paper is to realize the function of the system to the flexibility and convenience of the control terminal. The system is based on the Android operating system to develop intelligent terminal control software with high practical value, simple operation, and convenient use [9, 10].

Its functional realization architecture diagram is shown in Figure 2.

According to user needs, this control software needs to achieve the following goals:

- It is simple and convenient to operate, and the interface is simple and beautiful.
- It is convenient for users to query environmental information, health information, and video information and can effectively remotely control the LED lights, FAN, and buzzer of the data acquisition terminal.
- It protects user privacy by setting passwords and setting up access cards.
- The system runs stably, safely, and reliably.

As can be seen from the functional architecture diagram, the main window of this control software includes four subwindows. An information query window is used to obtain information, and Appliance control window is used for remote control. The System Setup window is used to receive information. Threshold settings are the logoff windows that are used to complete the logoff feature.

#### 3.1.3. Smart Watch

Smartphones are very useful if the patient is the elderly and children. The elderly move slowly, and when they fall, they cannot immediately use their mobile phones to call for help. But if they are wearing a smartwatch, it is easier to ask for help. Children are less vulnerable, smartphones are easily stolen or lost, and they are not easy to carry around. Therefore, wearing a smart watch on the wrist is a sensible choice for children's parents. For ordinary smartphone users, when the mobile phone is not around or in a bag, and the mobile phone mode is silent or vibrating, it is not easy to detect incoming calls or text messages, and there will be missed calls. In the case of an important call, this can have serious consequences. If people wear a smart watch, the watch can be associated with the mobile phone. It can receive the corresponding data information in real time, which is convenient and easy to operate [11]. For exercisers, mobile phones are inconvenient to carry and use during exercise. If it is replaced by a smart watch, it is not only easy to carry but also can check the time, listen to music, answer calls, etc. Therefore, the wide application of smart watches is a product of the times and a development trend.

*(1) Smart Watch Operating System.* At this stage, the main operating systems of smart watches on the market are divided into the following categories. They are Apple's Apple Watch, Samsung's Tizen, LG's Web OS, Pebble Technology's Pebble, Android-specific Android wear, and the Android native ecosystem [12]. The advantages and disadvantages of these operating systems mainly include the following aspects (Table 1).

Through the information in Table 1, it is found that the operating systems of various smart watches have different advantages and disadvantages. In view of the expansibility, ease of development, and ease of operation of the Android system, the research in this paper will be based on the Android operating system. On the basis of the Android operating system, the research and development and innovation of the health monitoring system are carried out [13].

*(2) Internal Structure of Android Smart Watch.* Observing the development process of smart watches, it can be seen that the traditional smart watch is to directly build the system in the smart phone into the watch. Information is presented through the watch display. This kind of smart watch is equivalent to a miniature smart phone. Until the last few years, Google has developed an operating system Android wear based on the Android system specifically for smart watches, which has aroused people's pursuit of wearable devices. From the perspective of market sales, the traditional Android smartwatch is not the main body. But there are also many domestic producers making such watches. The disappearance of such watches will take some time. During this period, users will also tend to use and buy the watch [14].

### 3.2. CYP1B1 Gene Polymorphism and Lung Cancer

The amino acid changes in the corresponding enzyme proteins caused by single nucleotide mutations (SNPs) of the CYP1B1 gene can cause differences in the susceptibility of different individual tumors by affecting the enzymatic reaction process related to the activation of carcinogens. So far, 167 SNPs of CYP1B1 have been discovered in humans. And many studies have focused on four SNPs such as rs10012 (R48G), rs1056827 (A119S), rs1056836 (L432V), and rs1800440 (N453S). In the past ten years, with the continuous development of human gene polymorphism research, the correlation between CYP1B1 and malignant tumors has also been deeply and widely studied. This has certain guiding significance for the prevention and treatment of malignant tumors. However, the specific mechanism of the involvement of CYP1B1 gene polymorphisms in the occurrence of malignant tumors has not yet been fully revealed [15].

#### 3.2.1. The Concept of CYP1B1 Gene Polymorphism

The CYP1B1 gene is located at 2p22.2 on the short arm of chromosome 2. DNA is about 12 kb in length and consists of 3 exons and 2 introns. Its mRNA size is 5.2 kb and encodes a protein consisting of 543 amino acids [16]. The current study found that there are 167 SNPs in CYP1B1. Among them, there are many studies on the relationship between gene polymorphism and cancer at 4 SNPs. They are (1) rs10012, codon 48 on exon 2: the codon CGG encoding arginine (Arg) at this site is replaced by the codon GGG of glycine (Gly), abbreviated as R48G. (2) rs1056827, codon 119 on exon 2: the codon GCC coding for alanine (Ala) at this site is replaced by the codon TCC for serine (Ser), which is abbreviated as A119S. (3) rs1056836, codon 432 on exon 3: the codon CTG encoding leucine (Lue) at this site is replaced by the codon GTG of valine (Val), abbreviated as L432V. (4) rs1800440, codon 453 on exon 3: the codon AAC encoding asparagine (Asn) at this site is replaced by the codon AGC of serine (Ser), which is abbreviated as N453S. In a study discussing the relationship between CYP1B1 gene polymorphisms and cancer, haplotype A accounted for the largest proportion (47%) in 60 lung cancer patients in NCI (National Cancer Institute, US National Cancer Center). Accordingly, lung cancer patients were divided into A/A type, A/X type, and X/X type.

#### 3.2.2. Lung Cancer

Lung cancer is one of the common primary malignant tumors of the respiratory system. With the modern unhealthy lifestyle, life rhythm, smoking, environmental pollution, and population aging, the incidence of lung cancer is increasing year by year. At present, the prevention and treatment of lung cancer is one of the important issues of worldwide concern. According to the survey report of the World Health Organization, lung cancer has gradually become the cancer with the highest incidence in recent decades. Lung cancer ranks first among all tumors. Currently, the clinical treatments for lung cancer include surgery, radiotherapy, chemotherapy, targeted therapy, immunotherapy, and multidisciplinary comprehensive therapy. Up to now, radical surgery for lung cancer is still the only possible way to cure lung cancer patients [17].

### 3.3. Data Mining Technology

#### 3.3.1. The Meaning of Data Mining Technology

Data mining refers to the process of searching out the information hidden in it through algorithms from a large amount of data. This is a step in the discovery of data knowledge. The methods used by data mining technology to achieve the above goals usually adopt the following methods: statistical and analytical processing, situation retrieval, machine learning, expert systems, and pattern recognition. The application of these methods is inseparable from the development of computer science [18].

The following describes several common methods of operation in data mining:

1. Neural network: for the problem of data mining, neural network is generally a more suitable solution. The reason is that it has some good properties, such as good robustness, parallel processing, distributed storage, self-organizing adaptability, and high fault tolerance. Different neural network models should be used for different data mining applications. For example, for data mining problems such as prediction, classification, and pattern recognition, it is more appropriate to use a feedforward neural network model. Neural network models also have an inconvenience, which is commonly referred to as “black box.” The learning and decision-making methods of the network throughout the process are difficult to understand and use [19].
2. Decision tree method: the idea of the decision tree method is to first classify a large amount of unordered data purposefully. Then, it seeks out those hidden and valuable information, which is usually used in the establishment of predictive models. Decision tree methods are not only quick to classify but also simple and clear to describe. But there are still some problems. It is a nonincremental learning algorithm. Decision trees are usually aimed at univariate data, and it is difficult to express complex concepts clearly. Interrelationships between the same sex are not sufficiently emphasized. Noise immunity is poor.
3. Statistical analysis method: in the database, there are two types of relationships between field items: functional relationship (a deterministic relationship that can be represented by a functional formula) and a correlation relationship (a certain related deterministic relationship, but cannot be represented by a functional formula).
4. Fuzzy set method: when using the fuzzy set method in practical problems, the intensity of fuzziness depends on the complexity of the system: when the complexity is low, the fuzziness is poor [20]. Commonly used fuzzy set methods mainly include fuzzy decision making, fuzzy pattern recognition, fuzzy evaluation, and fuzzy clustering analysis.

#### 3.3.2. Artificial Neural Network Modeling

Artificial neural network (ANN) is a technology that simulates human intelligent behavior. The input layer is composed of multiple neurons, which can accept a large amount of nonlinear input information. This input information are called input vectors. In the output layer, information goes through a series of transmission, analysis, and trade-offs in the connections between neurons. The structure of the operation model of neural network is mainly divided into two parts: a large number of nodes and the connection part between nodes. Each node in the network represents a specific output function (also called an excitation function). The connection between each two nodes represents a weighted value (also called weight) for the signal passing through this connection. Since the composition, connection method, weighting value, and output function of each network are different, the final output of the network is also different. Its model is shown in Figure 3.

Artificial neural networks can be classified from different perspectives (network performance, structure, learning methods, etc.). Taking the common multilayer structure forward network as an example, the network consists of 3 parts: input layer, hidden layer, and output layer.

#### 3.3.3. BP Neural Network Theory

The neural units on the same layer of the BP neural network are not connected to each other. The layers are connected to each other, generally in a fully connected way. The entire network is one-way propagation. The structure of the 3-layer BP neural network commonly used is shown in Figure 4 [21].

The learning process and steps of BP network are as follows:

(1) It draws random values on the interval (−1, 1) and assigns each of the weights *Q*_*ij*_ and *D*_*js*_, and thresholds *δ*_*j*_ and *χ*_*s*_.
(2) It randomly selects a set of input and target samples *L*_*r*_=(*A*_1_^*r*^, *A*_2_^*r*^, ⋯, *A*_*v*_^*r*^) and *S*_*r*_=(*B*_1_^*r*^, *B*_2_^*r*^, ⋯, *B*_*m*_^*r*^), provides them to the network, uses the input *A*_*i*_, the threshold *δ*_*j*_, and the connection weight *Q*_*ij*_ to calculate the input *T*_*j*_ of each neural unit on the hidden layer, and then calculates the output *K*_*j*_ according to the transfer function. The formula is as follows:
  (1) $$\begin{array}{c} T_{j}=\overset{v}{\underset{i=1}{\sum }}A_{i}Q_{ij}+\delta_{j},\\ K_{j}=g\left(T_{j}\right)\text{.} \end{array}$$
(3) It calculates the input *H*_*s*_ of each neural unit on the output layer according to the output *K*_*j*_ of the hidden layer, the connection weight *D*_*js*_, and the threshold *χ*_*s*_. It then calculates the output *c*_*s*_ according to the transfer function. The calculation formula is as follows:
  (2) $$\begin{array}{c} H_{s}=\overset{p}{\underset{j=1}{\sum }}K_{j}D_{js}+\chi_{s},\\ c_{j}=g\left(H_{s}\right)\text{.} \end{array}$$
(4) It calculates the generalized error *J*_*s*_^*r*^ of each unit on the output layer according to the target vector *S*_*r*_ and the actual output *C*_*s*_ of the network. The formula is as follows:
  (3) $$\begin{array}{c} J_{s}^{r}=\left(B_{s}^{r}-C_{s}\right)•C_{s}•\left(1-C_{s}\right)\text{.} \end{array}$$
(5) It calculates the generalized error *E*_*j*_^*r*^ of each unit on the hidden layer based on the output *K*_*j*_ on the hidden layer, the generalized error *J*_*s*_^*r*^ on the output layer, and the connection weight *D*_*js*_. The formula for calculation is as follows:
  (4) $$\begin{array}{c} E_{j}^{r}=\left(\overset{m}{\underset{s=1}{\sum }}J_{s}^{r}•D_{js}\right)•K_{j}•\left(1-K_{j}\right)\text{.} \end{array}$$
(6) It modifies the threshold *χ*_*s*_ and connection weight *D*_*js*_ according to the output *K*_*j*_ of each unit on the hidden layer and the generalized error *J*_*s*_^*r*^ of each unit on the output layer.
  (5) $$\begin{array}{c} D_{js}\left(V+1\right)=D_{js}\left(V\right)+\alpha •J_{s}^{r}•K_{j},\\ \chi_{s}\left(V+1\right)=\chi_{s}\left(V\right)+\alpha •J_{s}^{r}\left(0<\alpha <1\right)\text{.} \end{array}$$
(7) It completes the correction of the connection weight *Q*_*ij*_ and the threshold *δ*_*j*_ according to the input *A*_*i*_ on each unit of the input layer and the generalized error *E*_*j*_^*r*^ on each unit of the hidden layer.
  (6) $$\begin{array}{c} Q_{ij}\left(V+1\right)=Q_{ij}\left(V\right)+\beta •E_{j}^{r}•\alpha_{i}^{r},\\ \delta_{j}\left(V+1\right)=\delta_{j}\left(V\right)+\beta •E_{j}^{r}\left(0<\beta <1\right)\text{.} \end{array}$$
(8) After completing the above training steps, the input samples are randomly selected and handed over to the network for repeated training operations until the training of all samples is completed. After the network training is completed, its convergence should also be judged. There is a preset minimum value for the global error *E* of the network. If the error after re-extracting a set of input samples and the corresponding target samples after training is less than the set error, then the network is converged. The learning times of the network are also set in advance. Once the number of learning times after training is larger than the set in advance, the training network cannot converge.

The learning process of the entire network mainly includes the above eight steps. After training, it is necessary to analyze and test the performance of the network. Before network training, the data have been divided into training set and test set. The data in the training set complete the training of the network. The data of the test set need to complete the test of the network. It randomly selects samples from the test set to input the network and tests the performance of the network by checking the classification results of the network. It should be noted that the learning samples of the network cannot have the exact same pattern as the test sample set. In this way, the performance of the network can be tested more accurately.

### 3.4. Basic Theory of Deep Learning and Target Detection Application Algorithms

#### 3.4.1. Basic Theory of Deep Learning

Deep neural network (DNN), convolutional neural network, deep belief network (DBN), and recurrent neural network (RNN) and other network frameworks are commonly used deep learning frame. Deep learning is a very popular method in machine learning, covering a wide range of theoretical perspectives. In order to achieve more intelligent human-computer interaction, researchers imitate the human brain and thinking. They build various neural network models, and deep learning is one of them. By creating a model to learn data features, finding a better data representation is the primary purpose of representation learning [22]. Deep learning has a wide range of applications, including computer vision, speech recognition, natural language processing, and bioinformatics. Among them, for computer vision, convolutional neural networks use convolution and pooling to effectively reduce the number of weight parameters. Even if it directly inputs multidimensional images, it will not cause huge computational burden. It then takes into account that convolutional neural networks are highly invariant to many forms of transformation, such as translation, angle, and scaling. The target detection algorithm designed in this paper is based on the convolutional neural network structure.

#### 3.4.2. The Basic Idea of Convolutional Neural Network

Figure 5(a) shows the connection method of traditional neural network—full connection. The local connection is shown in Figure 5(b). Compared with the fully connected network, the locally connected approach reduces the number of weight parameters exponentially.

#### 3.4.3. Basic Structure of Convolutional Neural Network

The convolutional neural network is a neural network that mainly consists of convolutional layers and contains various types of network layers. Its basic structure is shown in Figure 6.

*(1) Convolutional Layer.* Convolution operations are divided into continuous convolution and discrete convolution. The formula for continuous convolution is as follows:

(7) $$\begin{array}{c} B\left(s\right)=\overset{\infty }{\underset{-\infty }{\int }}A\left(p\right)J\left(s-p\right)dp=A\left(s\right)•J\left(s\right)\text{.} \end{array}$$

The discrete convolution formula is as follows:

(8) $$\begin{array}{c} B\left(m\right)=\overset{\infty }{\underset{-\infty }{\sum }}A\left(i\right)J\left(m-i\right)=A\left(m\right)•J\left(m\right)\text{.} \end{array}$$

The convolution operation of the convolutional neural network belongs to the discrete convolution operation. Moreover, it is somewhat different from the definition in analytical mathematics, and it is a linear operation. The formula is expressed as follows:

(9) $$\begin{array}{c} g\left(A,B\right)•\omega \left(A,B\right)=\overset{v}{\underset{k=-v}{\sum }}\overset{c}{\underset{s=-c}{\sum }}\omega \left(k,s\right)g\left(A-k,B-s\right). \end{array}$$

In the formula, *g*(*A*, *B*) is the gray value of row *A* and column *B* in the image; *ω*(*A*, *B*) is convolution kernel or filter.

*(2) Downsampling Layer.* The algorithm expression for average downsampling is as follows:

(10) $$\begin{array}{c} K_{ij}=\frac{\left(\overset{d}{\underset{i=1}{\sum }}\overset{d}{\underset{j=1}{\sum }}G_{ij}\right)}{d^{2}}+c^{2}\text{.} \end{array}$$

The algorithm expression for maximum downsampling is as follows:

(11) $$\begin{array}{c} K_{ij}=\max_{i=1,j=1}\left(G_{ij}\right)+c_{2.} \end{array}$$

In the formula, *G* is feature map matrix; *K* is the obtained downsampling feature map; *d* is movement step; $\max_{i=1,j=1}\left(G_{ij}\right)$ is the largest element taken from the region of size dxd in the input feature map *G*.

*(3) Logistic Regression and Softmax Layer.* The logistic regression algorithm is a classification algorithm. The range of output values is as follows:

(12) $$\begin{array}{c} 0\leq J_{\theta }\left(A\right)\leq 1\text{.} \end{array}$$

It is suitable for the case where the value of label *B* is discrete, such as 0, 1, 1, and 0. We suppose that

(13) $$\begin{array}{c} J_{\theta }\left(A\right)=f\left(\theta^{s}A\right)\text{.} \end{array}$$

In the formula, *A* is eigenvector and *f* is logical function.

A commonly used logistic function is the sigmoid function, and the formula is as follows:

(14) $$\begin{array}{c} f\left(z\right)=\frac{1}{\left(1+e^{-z}\right)}\text{.} \end{array}$$

## 4. Experiment of Intelligent Health Monitoring Application

### 4.1. Software Test Results

It tests the system android-side software program according to the above-mentioned process, and also adopts 3 rounds of 18 groups of data testing methods. The mobile phone client program sequentially obtains the physical information data transmitted by the underlying information collection boards, and compares it with the data measured by the medical physical equipment. The data show good results with small deviations. The following are several groups of examples of information comparison, as shown in Tables 2 and 3.

It can be seen from Tables 2 and 3 that the information data values displayed by the android software have a high degree of matching with the measured values, and the data consistency is strong. In the table, the physical measurement temperature was 37.2°C at the 5th second, the software read value was 37°C, the pulse was 81 times per minute, and the software read value was 81.5 times per minute, and the data difference was small. At the same time, the software interface is neat and beautiful, simple and easy to use, and convenient for finger touch. After many tests, the program runs well without bugs. Therefore, the system android software meets the requirements and the test passes.

### 4.2. Implementation of Apriori Algorithm

The steps of using the algorithm for data mining are as follows: it first codes the system software and assigns some controls to variable values, such as setting the temperature control as a temperature count variable. It calculates and processes the data of the number of clicks and the time interval of the control, stores the statistical results in the database, and then transmits it to the cloud server. After the server receives the data, it uses the Apriori algorithm to analyze and summarize the user's behavior, form a corresponding evaluation report, and provide the user with a personalized functional mode. In fact, network data mining technology is also carried out in this way. It extracts preference data from the user's browsing history and stores the user's browsing log records. It arranges the display graph, highlighting data with strong correlations (Figure 7). It applied intelligent health monitoring to a study to observe four patients after minimally invasive surgery for lung cancer, and the four patients were *A*, *B*, *C*, and *D*.

### 4.3. Health Monitoring System Data Results

For the data analysis of the health monitoring system, this experiment used the Apriori algorithm and the QlikView analysis tool to form a visual chart. The details are shown in Figure 8.  Figure 8(a) uses body temperature monitoring data and user personal information data to count the relationship between users and temperature measurements.  Figure 8(b) correlates the monitored weight data with the individual situation of the user for analysis and research. From the analysis of many data, the user's preference for certain functions of the system can be concluded. By calculating the number of times user *C* measures body temperature and weight, height, blood type, and other data, C's behavior can be analyzed and predicted. This can push the appropriate information to the user.

Figure 8 mentioned the number of clicked controls and the analysis of individual user associations, and then studied the relationship between users and time intervals. It uses the Apriori algorithm to analyze the time nodes of user operations. The main steps are divided into the following aspects. First, it divides behavioral time into unequal parts. It is generally in the morning, noon, afternoon, evening, early morning, and other time stages. Second, it analyzes and counts the behavior of users through different time periods. Third, it summarizes the statistical results. Then, the user's number of clicks on the control and the use of time interval are integrated to form a more comprehensive and complete analysis and research, so as to obtain accurate user preferences and usage frequencies of the system.

The user's body temperature measurement data and time are correlated and analyzed. This time period can be divided into days, weeks, and months. In each time period, the number of users using body temperature measurement is analyzed and counted. When using the body temperature measurement continuously for one day, it can be preliminarily inferred that the user's body has deteriorated according to the measured body temperature data. Then, the system launches some reminders based on the local climate and user behavior on that day.

When the relationship between the user's weight value and the time is detected, the time may be divided into two-hour intervals. Then, it analyzes and counts the user usage in each time period, determines the duplicate item sets in each time period, and performs several more times until the item set with the highest repetition is determined. This design is similar to RFID supply chain data analysis techniques in time series. According to the monitored data, user *C* likes to use the system to measure body weight before and after meals, and most people do so during this time period. Therefore, when an optimized weight measuring instrument appears, the system can automatically push relevant information to the user. However, there are not many test data used, and the obtained analysis effect is not very scientific, and further research is needed.

## 5. Discussion

With the development of economy and the improvement of people's material living standards, intelligent health monitoring stations based on information and intelligence have emerged. The development of sensor technology also provides more accurate health data for intelligent monitoring, enabling people to detect important physiological indicators without leaving home [23].

In this paper, the overall functional architecture of the system is designed according to the market hardware performance and the needs of users. It explains each functional module in detail, formulates the program flow chart, and realizes the research and development of the system in combination with the software and hardware of system. A health monitoring system based on a smart watch can monitor the user's body temperature and weight data. The system analyzes the data through corresponding programs and gives appropriate recipes and exercise suggestions. It allows people to enhance the concept of sports and ensure the quality of life. Then, the data of the system are analyzed, using the theory of data mining. It applies the Apriori algorithm to the application design of the system. It also briefly describes the practical application and steps of the Apriori algorithm in the health monitoring system, and forms a corresponding evaluation report.

Limited by my time and ability, there are still some areas for improvement in this research. The intelligent health monitoring system designed only to monitor human body temperature and weight data, store and transmit data to the server, browse historical data, and analyze the received data from the server. It forms a corresponding evaluation report and returns it to the mobile terminal to provide users with some recipes and suggestions for exercise methods. There is no detailed elaboration and research on how the cloud server operates and processes data. It also lacks other health data to fully analyze the user's health.

## 6. Conclusions

The intelligent health monitoring system based on this study is generated based on people's attention to the mobile health system. With the improvement of living standards, people pay more and more attention to health. Mobile health monitoring systems have become the focus of intelligent research and medical research. It also uses smart wearable devices and network transmission technology to research and develop this intelligent health monitoring system. Accurate human body temperature and weight data can be obtained through this system, and the collected data are transmitted to the cloud server. The server analyzes and summarizes the received data, and forms a corresponding evaluation report. It is displayed through the mobile phone or watch client. Users can browse the history of body temperature and weight through the smartphone client. The server analyzes and processes the monitoring data, provides users with healthy recipes and suggestions on exercise methods, and ensures the user's quality of life and physical health. Moreover, global variables are set for the controls in the system, and it records the usage of each control by the user through clicking the button. It analyzes the user's behavior and preferences, and then pushes appropriate information to the user and performs future system updates.

## Figures and Tables

**Figure 1:** Overall design of the system.

**Figure 2:** Control terminal functional architecture diagram.

**Figure 3:** Neural network model.

**Figure 4:** Structure diagram of 3-layer BP neural network.

**Figure 5:** Fully connected neural network and partially connected neural network. (a) Fully connected neural network. (b) Locally connected neural network.

**Figure 6:** Deep convolutional neural network architecture.

**Figure 7:** Apriori core algorithm.

**Figure 8:** User temperature/weight measurement viscosity from January to March. (a) User temperature experimental value. (b) Experimental value of user weight.

**Table 1:** Comparison of advantages and disadvantages of smart watch systems.

Operating system	Application company	Advantage	Shortcoming
Apple watch	Apple Inc	Fluency, introduction, stability, and beauty	No open source and poor customization

Tizen	Samsung	Stability and flexibility	No open source and no support for Chinese

Pebble	Pebble	Compatible with Android, iOS smartphone, and long standby time	Insensitive response

Web OS	HP, LG	Easy to use, open source, and beautiful	Not widely used and poor user experience

Android customized system	Nutshell, Sony, Samsung, M0T0360, and Huawei	Open source, smooth, concise, and beautiful	Inaccurate speech recognition and short endurance

Android original ecosystem	Ingenic	Open source, insert sim card, make phone calls, send text messages, connect WiFi, Bluetooth, etc.	Google software vulnerability

**Table 2:** Comparison between software display data and measured data (temperature).

Time/s temperature (°C)	Physical measured value	Software read value
0	36.7	36.7
5	37.2	37
10	36.8	36.8
15	36.9	36.9
20	37.1	37.11
25	37	37.02
30	37.2	37.2
35	37.1	37.1
40	37.2	37.2
45	37.3	37.32
50	37.5	37.5

**Table 3:** Comparison between software display data and measured data (pulse).

Time/s pulse (times/minute)	Physical measured value	Software read value
0	83	83
5	81	81.5
10	79	79.9
15	80	80
20	77	77
25	79	78.9
30	77	77
35	76.5	76.5
40	77	77
45	75.5	75.4
50	80.5	80.5

## Data Availability

No data were used to support this study.
